The article "Radiological findings in low-dose CT for COVID-19 pneumonia in 182 patients: Correlation of signs and severity with patient outcome" was published in 2022. Journal: Medicine (Baltimore).

# Radiological findings in low-dose CT for COVID-19 pneumonia in 182 patients: Correlation of signs and severity with patient outcome

**DOI:** 10.1097/MD.0000000000028950

**Published:** 2022-03-04

**Authors:** Charlotte M. BiebaÛ, Jeroen N. Desmet, Adriana Dubbeldam, Lesley Cockmartin, Walter M. Coudyzer, Johan Coolen, Johny A. Verschakelen, Walter De Wever

**Affiliations:** 1 Department of Radiology, University Hospitals Leuven, Leuven, Belgium.

**Keywords:** COVID-19, diagnosis, disease progression, tomography, triage, X-ray computed

## Abstract

To characterize computed tomography (CT) findings of coronavirus disease 2019 (COVID-19) pneumonia and their value in outcome prediction.

Chest CTs of 182 patients with a confirmed diagnosis of COVID-19 infection by real-time reverse transcription polymerase chain reaction were evaluated for the presence of CT-abnormalities and their frequency. Regarding the patient outcome each patient was categorized in 5 progressive stages and the duration of hospitalization was determined. Regression analysis was performed to find which CT findings are predictive for patient outcome and to assess prognostic factors for the hospitalization duration.

Multivariate statistical analysis confirmed a higher age (OR = 1.023, *P* *=* *.025*), a higher total visual severity score (OR = 1.038, *P* *=* *.002*) and the presence of crazy paving (OR = 2.160, *P* *=* *.034*) as predictive parameters for patient outcome. A higher total visual severity score (+0.134 days; *P* *=* *.012*) and the presence of pleural effusion (+13.985 days, *P* *=* *0.005*) were predictive parameters for a longer hospitalization duration. Moreover, a higher sensitivity of chest CT (false negatives 10.4%; true positives 78.6%) in comparison to real-time reverse transcription polymerase chain reaction was obtained.

An increasing percentage of lung opacity as well as the presence of crazy paving and a higher age are associated with a worse patient outcome. The presence of a higher total visual severity score and pleural effusion are significant predictors for a longer hospitalization duration. These results are underscoring the value of chest CT as a diagnostic and prognostic tool in the pandemic outbreak of COVID-19, to facilitate fast detection and to preserve the limited (intensive) care capacity only for the most vulnerable patients.

**Key points**

- Computed Tomography helps clinicians in triage of patients suspicious for COVID-19 pneumonia.
- Retrospective study shows that Chest Computed Tomography provides greater diagnostic confidence for detection of COVID-19 infection.
- Chest CT findings can be used to predict the outcome in COVID-19 patients.

The article "Radiological findings in low-dose CT for COVID-19 pneumonia in 182 patients: Correlation of signs and severity with patient outcome" was published in 2022. Journal: Medicine (Baltimore).

## 1 Introduction

In December 2019 in Wuhan province, China, first reports were made of an outbreak of a new respiratory virus, now known as the highly contagious severe acute respiratory syndrome coronavirus 2 . On January 30, 2020, the World Health Organization declared this ongoing outbreak as a global public health emergency. On March 11, 2020 it was reclassified as a global pandemic outbreak.

According to current insights in the literature, the characteristic radiological presentation of coronavirus disease 2019 (COVID-19) pneumonia is that of bilateral distribution of ground-glass opacities (GGO), with or without consolidation, mostly affecting the basal and peripheral lungs.^[1]^ However, upon further analysis, a diversity of computed tomography (CT) findings were found,^[1]^ and the CT-appearance of COVID-19 pneumonia is depending on the time between symptom onset and the CT scan.^[2]^

The Fleischner Society Statement on Chest Imaging and COVID-19 stated that chest CT is indicated in patients with COVID-19 who have worsening respiratory status or for medical triage of patients with suspected COVID-19 who present with moderate to severe clinical features and a high pretest probability of COVID-19 pneumonia.^[3]^ In accordance with the Fleischner Society Statement on Chest Imaging and COVID-19, we used low-dose chest CT as a triage system, in correlation with clinical parameters (saturation%, dyspnoea) to assess the risk for disease progression in patients with moderate to severe clinical features and to evaluate the need for hospitalization, intensive care unit (ICU), and/or intubation in COVID-19 pneumonia. In this pandemic outbreak, fast diagnosis and the detection of high-risk patients with a worse prognosis are crucial but challenging. The aim of this study was to evaluate the value of chest CT scan as a diagnostic and prognostic tool in the triage system for patients with COVID-19 pneumonia to determine which patients needed to be hospitalized or admitted to the ICU.

## 2 Material and methods

### 2.1 Study design

The retrospective analysis was approved by the Ethics Committee Research UZ/KU Leuven. Written informed consent was waived by the Institutional Review Board. Between March 21, 2020 and April 11, 2020, 763 patients underwent RT-PCR and noncontrast low-dose chest CT scan. In 182 patients, RT-PCR was positive for COVID-19 and CT was performed before or within a time interval of 4 days of the RT-PCR; patients with a positive RT-PCR in a time interval of more than 4 days after the index CT were excluded because of the possible later onset of the infectious disease.

### 2.2 Study implementation

All CT examinations were performed on a 128 detector-row CT scanner (Siemens Definition Flash, Forchheim, Germany) with a single breath hold. A noncontrast low-dose protocol was performed with the following parameters (gantry speed of 0.5 seconds per rotation, slice collimation: 128 × 0.6 mm, pitch factor 1.2, slice thickness 1 and 3 mm, slice increment 0.7 and 3 mm), except for mAs and kV settings depending on patient weight (<50 kg: 80 kV and 30 mAs; 50–80 kg: 120 kV and 20 mAs; >80 kg: 140 kV and 28 mAs).

The article "Radiological findings in low-dose CT for COVID-19 pneumonia in 182 patients: Correlation of signs and severity with patient outcome" was published in 2022. Journal: Medicine (Baltimore).

Chest CT scans were evaluated for CT findings and their frequency by 4 experienced thoracic radiologists. Typical CT findings described for COVID-19 include GGO, consolidations, crazy-paving pattern, subpleural reticulation, air bronchogram, (reversed) halo sign, subpleural bands, vascular dilatation, focal pleural thickening, and airway changes.^[1]^ Examples of atypical CT findings are centrilobular nodules, tree-in-bud pattern, enlarged lymph nodes, pleural effusion, and cavitation.^[1]^

For estimating the severity, a visual scoring of the lung injury per lobe in 5 categories was used (0: no involvement, 1: 0%–5% involvement, 2: 5%–25% involvement, 3: 25%–50% involvement, 4: 50%–75% involvement, 5: >75% involvement).

Regarding the patient outcome, each patient was categorized in the highest achieved stage of 5 progressive stages (quarantine at home, admission to a non-ICU, admission to the intensive care unit, intubation at the intensive care unit, and mortality) and the duration of hospitalization was determined.

### 2.3 Statistical analysis

Ordinal logistic regression (univariate and multivariate) analysis was performed to find which CT findings of COVID-19-positive patients are predictive for patient outcome and linear regression analysis was performed to assess prognostic factors for the hospitalization duration. The cutoff value for the parameters visual score of lung opacity and age associated with the worst patient outcome (deceased) was determined by the Youden's index on the receiver-operator characteristic curve. Similarly, the cutoff value for the visual score of lung opacity associated with a hospitalization duration longer than the mean of 11 days was determined. Statistical analysis was performed using the IBM Statistical Package for Social Sciences (SPSS version 13, IBM Corp, Armonk, NY); statistical significance level was 0.05.

## 3 Results

### 3.1 Patient characteristics

Of 763 patients with CT and RT-PCR, 182 (23.9%) COVID-19-positive patients could be included with a summary of the patient characteristics listed in Table 1. In the study group there were slightly more men (60.4%) in comparison with women (39.6%) affected by COVID-19 pneumonia and the median age was 65 years. The need for admission to a non-ICU was 84.6%, for admission to an ICU 25.8% and for intubation at the ICU 14.9% with an overall mortality rate of 11.5%.

The article "Radiological findings in low-dose CT for COVID-19 pneumonia in 182 patients: Correlation of signs and severity with patient outcome" was published in 2022. Journal: Medicine (Baltimore).

**Table 1:** Summary of patient characteristics (n = 182).

Parameter	n (%)	Parameter	n (%)
Sex		Symptoms	
Men	110 (60.4)	Fever	134 (73.6)
Women	72 (39.6)	Cough	108 (59.3)
Age (yr)		Dyspnoea	135 (74.2)
Mean	65	Myalgia	23 (12.6)
Standard deviation	16.22	WBC count 10^9^/L (ref 4–10.00)	
Range	22–91	Mean	6.71
Smoking		Standard deviation	4.46
Active smoker	10 (5.5)	Range	<0.10–281.67
Ex-smoker	61 (33.5)	Lymphocyte count 10^9^/L (ref 1.2–3.6)	
Nonsmoker	88 (48.4)	Mean	1.06
Unknown status	23 (12.6)	Standard deviation	0.79
BMI		Range	0–277
Mean	27.4	CRP mg/dL (ref. <5.0)	
Standard deviation	0.47	Mean	76.25
Range	10.8–47.1	Standard deviation	69.79
Outcome		Range	<0.3–441.1
No admission	28 (15.4)	Duration of hospitalization	
Admission to a non-ICU	154 (84.6)	Mean	11.15
Admission to ICU	47 (25.8)	Standard deviation	0.78
Admission to ICU and intubated	29 (15.9)	Range	0–44
Mortality	21 (11.5)		

BMI = body mass index, CRP = C-reactive protein, ICU = intensive care unit, WBC = white blood cells.

### 3.2 CT performance

Chest CT examination was reported in 78.6% (143/182) as consistent, in 11.0% (20/182) as inconclusive, and in 10.4% (19/182) as inconsistent for COVID-19 pneumonia.

### 3.3 Chest CT characteristics

The occurrence rates of typical, atypical, and rare CT findings for COVID-19 pneumonia as well as the distribution pattern and total visual score of lung injuries are described in Table 2. Bilateral lung involvement was observed in 95.1% and multilobular involvement in 93.4%. The left lower lobe was most frequently involved (96.7%), followed by the right lower lobe (95.1%), the both upper lobes (87.9%), and “least” frequent in the right middle lobe (80.8%). Most often there was a peripheral-central distribution with peripheral predominance (62.1%). The predominant peripheral and basal distribution may be due to the fact that the endobronchial spreading virus invades bronchioles and alveoli, causing bronchiolitis and subsequently inflammatory reactions in the alveoli and interstitium (airspace filling and interstitial thickening) which needs the participation of blood vessels and lymphatics who are more abundant in the peripheral and lower areas of the lungs as reported in earlier studies.^[4,5]^ The large airways are less affected by the virus due to its better viral clearance (abundant cilia and strong immune function).^[5]^ In 2.2% no alterations on chest CT were reported and 17% demonstrated with a mildly/early stage of the disease with only peripheral and predominantly basal opacities.

The article "Radiological findings in low-dose CT for COVID-19 pneumonia in 182 patients: Correlation of signs and severity with patient outcome" was published in 2022. Journal: Medicine (Baltimore).

**Table 2:** Summary of chest CT characteristics (n = 182).

Finding				n (%)		Finding	n (%)
**Involvement**						**Typical findings**	
Bilateral				173 (95.1)		Ground-glass opacities (GGO)	177 (97.3)
Multilobular				170 (93.4)		Nodular GGO	152 (83.5)
Frequency of lobe involvement						Focal pleural thickening^1^	160 (87.9)
Right upper lobe				160 (87.9)		Calcified plaques	10 (5.5)
Right middle lobe				147 (80.8)		Subpleural bands^2^	155 (85.2)
Right lower lobe				173 (95.1)		High opacities	152 (83.5)
Left upper lobe				160 (87.9)		Round opacities	74 (40.7)
Left lower lobe				176 (96.7)		Linear opacities	141 (77.5)
**Distribution pattern**						Bronchial wall thickening	130 (71.4)
Peripheral				31 (17.0)		Calcified	50 (27.5)
Peripheral-central				147 (80.8)		Vascular dilatation	91 (50.0)
Peripheral predominance				113 (62.1)		Subpleural reticulation	66 (36.3)
Central				0 (0)		Halo sign	39 (21.4)
No lung involvement				4 (2.2)		Crazy-paving	34 (18.7)
**Visual scoring n (%)**						Air bronchogram	31 (17.0)
	LUL	LLL	RUL	RML	RLL	**Atypical findings**	
0: 0% involvement	22 (12.1)	6 (3.3)	22 (12.1)	35 (19.2)	9 (4.9)	Centrilobular nodules	51 (28.0)
1: 0-5%	77 (42.3)	58 (31.9)	80 (44.0)	80 (44.0)	53 (29.1)	Enlarged lymph nodes	29 (15.9)
2: 5-25%	49 (26.9)	62 (34.1)	41 (22.5)	40 (22.0)	60 (33.0)	Pleural effusion	24 (13.2)
3: 25-50%	26 (14.3)	41 (22.5)	24 (13.2)	21 (11.5)	42 (23.1)	Tree-in-bud pattern	4 (2.2)
4: 50-75%	8 (4.4)	11 (6.0)	11 (6.0)	4 (2.2)	12 (6.6)	Cavitation	0 (0)
5 :> 75%	0 (0.0)	4 (2.2)	4 (2.2)	2 (1.1)	6 (3.3)	**Rare findings**	
						Bronchiectasis	18 (9.9)
						Pre-existing	7 (3.8)
						Reversed halo (atoll) sign	6 (3.3)
						Pneumothorax	2 (1.1)
						Cysts	1 (0.5)

GGO = ground-glass opacities, LLL = left lower lobe, LUL = left upper lobe, RLL = right lower lobe, RML = right middle lobe, RUL = right upper lobe.

Ground-glass opacities were reported in 97.3%, consolidations (Fig. 1A) in 83.5%, and bronchial wall thickening in 71% of cases. In the ground-glass opacities, a prominent central vascular structure was noted in 50% of cases and described as vascular dilatation. The subtle focal pleural thickening (Fig. 1B, 88%), subpleural bands (Fig. 1C, 85%), and subpleural reticulation (36%) are frequently present, confirming the “organizing pneumonia-like” aspect of COVID-19 pneumonia. In the late stage of the disease, the repair of the lung injury was presumed to be accompanied by the formation of organization with straight edges of the consolidation areas, subpleural alterations, and bronchiectasis. Centrilobular nodules are reported in 28% (Fig. 1D), tree-in-bud pattern in 2%, enlarged lymph nodes in 16% (Fig. 1E), and pleural effusion in 13% (Fig. 1F). The presence of enlarged lymph nodes, pleural effusion, and/or clustered centrilobular nodules may suggest bacterial superinfection.^[1]^

The article "Radiological findings in low-dose CT for COVID-19 pneumonia in 182 patients: Correlation of signs and severity with patient outcome" was published in 2022. Journal: Medicine (Baltimore).

**Figure 1:** Top 3 typical and atypical CT findings. A, Nodular ground-glass opacity: appearance of a hazy nodular ground-glass opacity (orange box), typically bilateral, and in the peripheral and lower parts of the lungs in COVID-19 pneumonia. B, Pleural thickening: adjacent to the peripheral opacities there is frequently a subtle focal pleural thickening confirming the “organizing pneumonia-like” aspect. C, Subpleural bands: axial CT image in a COVID-19 positive patient shows subpleural bands (yellow arrows) basal in the lung. Subpleural bands are defined as thin curvilinear opacities (1–3 mm thickness) lying subpleural and parallel to the pleural surface. Centrilobular nodules (D), enlarged lymph nodes (E), and pleural effusion (F) are the top 3 atypical CT findings: superimposed aspiration pneumonia in a COVID-19-positive patient with known CPFE (centrilobular emphysema and combined systemic sclerosis/scleroderma-related fNSIP). Axial CT image shows peripheral areas of ground-glass opacity and some clustered centrilobular nodules (red box) basal in the right lung. The mediastinal window shows enlarged mediastinal lymph nodes (blue arrows) and a small pleural effusion (purple arrow) basal in the right lung. The combined findings of nodules, enlarged lymph nodes, and pleural effusion are suggestive for bacterial superinfection. COVID-19 = coronavirus disease 2019, CT = computed tomography.

### 3.4 Statistical analysis

Each of the CT findings in Table 2 was evaluated by means of an ordinal logistic regression analysis and linear regression analysis to assess which CT findings are predictive for respectively patient outcome and hospitalization duration. The complete results are demonstrated in Tables 3 and 4.

**Table 3:** Ordinal regression univariate and multivariate analysis to find significant influencing CT characteristics on patient outcome.

Univariate ordinal regression analysis				
	OR	95% CI	Wald χ2 (1)	*P*
Visual score of lung opacity	1.058	1.039–1.076	39.369	<.0001^∗^
Bilateral lung pathology	6.931	1.956–24.582	8.998	.003^∗^
Multilobular lung pathology	4.860	1.659–14.253	8.305	.004^∗^
GGO	3.227	0.595–18.084	1.857	.173
Nodular GGO	0.680	0.330–1.402	1.092	.296
Consolidation	1.725	0.808–3.677	1.988	.159
Round opacities	1.423	0.820–2.472	1.570	.210
Linear opacities	1.756	0.899–3.432	2.712	.100
Nodules	1.134	0.619–2.077	0.166	.684
Halo sign	0.791	0.411–1.520	0.494	.482
Vascular dilatation	1.234	0.717–2.125	0.576	.448
Subpleural bands	1.020	0.476–2.186	0.003	.960
Bronchial wall thickening	4.104	1.039–16.200	4.060	.044^∗^
Bronchial wall calcifications	1.480	0.792–2.762	1.512	.219
Prior lung disease	1.297	0.628–2.678	0.496	.482
Tree-in-bud pattern	1.223	0.196–7.629	0.046	.830
Cavitations	–	–	–	–
Enlarged lymph nodes	4.166	2.002–8.680	14.540	<.0001^∗^
Air bronchogram	2.675	1.307–5.474	7.257	.007^∗^
Crazy paving	4.446	2.342–8.440	20.8	<.0001^∗^
Pleural effusion	4.191	1.912–9.189	12.808	<.0001^∗^
Pleural thickening	1.808	0.784– 4.166	1.929	.165
Pleural calcifications	1.790	0.166–1.885	0.880	.348
Pneumothorax	0.530	0.037–7.546	0.219	.640
Pulmonary embolism	2.361	0.473–11.787	1.096	.295
Subpleural reticulation	1.127	1.980 – 0.642	0.174	.677

Multivariate ordinal regression analysis				
	OR	95% CI	Wald χ2 (1)	*P*
Visual score of lung opacity score	1.038	1.014–1.062	10.010	.002^∗^
Bilateral lung pathology	2.105	0.787–12.346	0.681	.409
Multilobular lung pathology	0.688	0.143–3.311	0.218	.641
Air bronchogram	1.616	0.724–3.597	1.371	.242
Crazy paving	2.160	1.060–4.386	4.506	.034^∗^
Pleural effusion	1.597	0.657–3.891	1.069	.301
Enlarged lymph nodes	1.422	0.603–3.236	0.700	.403
Bronchial wall thickening	1.112	0.236–5.236	0.018	.893
Age	1.023	1.003–1.044	5.042	.025^∗^
Gender	1.198	0.653–2.199	0.340	.560
Dyspnea	1.664	0.829–3.333	2.046	.153

Ordinal regression analysis with patient outcome as dependent variable						
	OR	95% CI	Wald χ2 (1)	*P*	Sensitivity%	Specificity%
Crazy paving	0.468	0.235–0.487	4.683	.030^∗^	38	76
Age	1.024	1.006–1.043	6.672	.010^∗^	95	57
Total visual severity	1.049	1.030–1.069	26.919	<.001^∗^	33	88

GGO = ground-glass opacities.

∗ means significant values.

The article "Radiological findings in low-dose CT for COVID-19 pneumonia in 182 patients: Correlation of signs and severity with patient outcome" was published in 2022. Journal: Medicine (Baltimore).

**Table 4:** Linear regression univariate and multivariate analysis to find significant influencing CT characteristics on hospital duration.

Univariate linear regression analysis					
	B (d)	Mean (d)	95% CI	Partial ŋ^2^	*P*
Visual score of lung opacity	0.271	1.739	0.195–0.348	0.215	<.0001^∗^
Bilateral lung pathology	8.632	11.632	2.011–15.252	0.036	.011^∗^
Multilobular lung pathology	8.838	11.838	3.222–14.455	0.051	.002^∗^
GGO	8.798	11.398	0.511–18.106	0.019	.064
Nodular GGO	−1.852	10.848	−2.281 to 5.986	0.004	.378
Consolidation	3.674	11.743	0.490–7.839	0.017	.083
Round opacities	2.946	12.880	0.151–6.043	0.019	.062
Nodules	−2.115	9.612	−1.338 to 5.568	0.008	.228
Crazy paving	7.407	16.63	4.068–10.746	0.097	<.0001^∗^
Reversed Halo sign	−0.332	10.833	−8.272 to 8.936	0.000	.939
Halo sign	−0.137	11.049	−3.543–3.817	0.000	.942
Vascular dilatation	2.994	12.693	0.056–6.044	0.021	.054
Subpleural bands	1.009	11.305	3.312–5.330	0.001	.646
Bronchiectasis	4.763	15.471	0.470–9.997	0.018	.074
Bronchial wall thickening	5.001	11.376	2.457–12.459	0.010	.187
Bronchial wall calcification	0.937	11.864	2.652–4.525	0.001	.607
Pleural thickening	1.771	11.380	2.847–6.389	0.450	.003^∗^
Pleural calcifications	0.789	11.900	5.952–7.530	0.000	.818
Prior lung disease	2.532	13.267	1.594–6.657	0.008	.228
Tree-in-bud pattern	0.669	10.500	9.808–11.147	0.000	.900
Cavitations	–	–	–	–	–
Enlarged lymph nodes	9.204	18.833	5.291–13.118	0.107	<.0001^∗^
Air bronchogram	3.317	13.903	0.743–7.376	0.014	.109
Pleural effusion	9.799	19.600	5.575–14.023	0.105	<.0001^∗^
Subpleural reticulation	−1.269	10.348	−1.926 to 4.464	0.003	.434
Pulmonary embolism	8.366	19.200	0.918–17.649	0.017	.077
Pneumothorax	−4.707	6.500	−10.012 to 19.426	0.002	.529

Multivariate linear regression analysis					
	B (d)	Mean (d)	95% CI	Partial ŋ^2^	*P*
Visual score of lung opacity	0.134	20.523	0.030–0.238	0.038	.012^∗^
Bilateral lung pathology	−9.017	20.523	−29.204 to 47.239	0.001	.642
Multilobular lung pathology	7.578	20.523	6.831–21.987	0.007	.301
Crazy paving	0.069	20.523	−19.253 to 19.390	0.000	.994
Pleural effusion	13.985	20.523	4.384–23.587	0.048	.005^∗^
Enlarged lymph nodes	8.972	20.523	1.574–19.518	0.017	.095
Age	0.029	20.523	−0.068to 0.125	0.002	.559

Linear regression analysis with hospitalization duration as dependent variable							
	B (d)	Mean (d)	95% CI	Partial ŋ^2^	*P*	Sensitivity%	Specificity %
Visual score of lung opacity	0.239		0.163–0.316	0.176	<.001^∗^	78	64
Pleural effusion	−6.819		−10.781 to 2.858	0.061	<.001^∗^	56	70

GGO = ground-glass opacities.

∗ means significant values.

The article "Radiological findings in low-dose CT for COVID-19 pneumonia in 182 patients: Correlation of signs and severity with patient outcome" was published in 2022. Journal: Medicine (Baltimore).

An increase of 1 unit (in %) of lung opacity and consolidation as well as the presence of multilobular and bilateral lung involvement, air bronchogram, bronchial wall thickening, crazy paving, pleural effusion, and enlarged lymph nodes are associated with a worse patient outcome by means of an univariate ordinal logistic regression model. In the multivariate analysis only a higher age, total visual severity score, and the presence of crazy paving were associated with a higher need for admission to an (non-) ICU, intubation as well as a higher mortality rate and showed to be independent predictive parameters (Table 3). The cutoff value for the parameters visual score of lung opacity and age associated with the worst patient outcome was respectively 54 and 67 years (Table 3).

Subsequently a significant longer hospital stay was obtained with a higher total visual severity score as well as the presence of bilateral lung pathology, multilobular lung pathology, pleural effusion, enlarged lymph nodes, and crazy paving in the univariate linear regression model. In the multivariate analysis only a higher total visual severity score and the presence of pleural effusion are significant predictors for a longer hospitalization duration and showed to be independent predictive parameters (Table 4). The cutoff value for the visual score of lung opacity associated with a hospitalization duration longer than the mean of 11 days was 38 (Table 4).

The article "Radiological findings in low-dose CT for COVID-19 pneumonia in 182 patients: Correlation of signs and severity with patient outcome" was published in 2022. Journal: Medicine (Baltimore).

## 4 Discussion

The higher rates in admission to a non-ICU/ICU, the need for intubation, and the overall mortality rate in comparison with other studies^[6]^ are probably caused by the biased patient cohort consisting of (mostly elderly) patients with a need for admission to the hospital. In earlier studies, some patient characteristics like heightened ACE2 expression, older age, Vitamin D deficiency, male gender, non-O blood group types, underlying comorbidities (diabetes, hypertension, cardiovascular disease, poorly controlled hypothyroidism, chronic obstructive pulmonary disease [COPD]), and host genetics are associated with a higher infection risk and/or worse outcome.^[7]^

In the proven COVID-19-positive patients, the occurrence rates of each category (conclusive, inconclusive, and inconsistent) are similar to earlier studies.^[8,9]^ The low degree of false negatives (10.4% inconsistent CTs) and the high degree of positive CTs (78.6% consistent CTs) are consistent with the reported higher sensitivity of chest CT scan in comparison with RT-PCR.^[1–10]^

Concerning the chest CT characteristics, the occurrence rates were difficult to compare with earlier studies because most published studies investigated the evolutive CT imaging features of COVID-19 pneumonia in time after symptom onset. In general, the study cohort contained patients in a moderately to advanced stage of COVID-19 pneumonia explaining the higher reported occurrence rate of bilateral and multilobular involvement, the lower only peripheral and basal involvement and the higher occurrence rate of GGO, consolidations, crazy paving, and signs of bacterial superinfection.^[1–5]^ The distribution pattern and the estimated involvement per lung lobe was similar compared with earlier studies.^[2–4]^

The significantly higher occurrence rate of bronchial wall thickening compared with other international studies,^[1]^ can be due to the higher age (50/182 demonstrated bronchial wall calcifications) or underlying comorbidities (e.g., COPD) of the study group; also, “pseudo” wall thickening caused by the incidental expiration phase of the Chest CT scan can cause an overestimation of bronchial wall thickening. Also, some of the bronchial wall thickening can be due to inflammatory damage of the bronchial wall by the endobronchial spreading disease who's more abundant in severe/critical patients.

The frequently reported finding of vascular dilatation may correspond to the reported vascular wall thickening and intraluminal thrombogenic material in the injured small lung vessels and the subsequently angiogenesis.^[11,12]^

The 3 most common typical CT findings in COVID-19 pneumonia are ground-glass opacities, subpleural bands, and a focal pleural thickening adjacent to the opacities (Fig. 1). Centrilobular nodules, pleural effusion, and enlarged lymph nodes are the 3 most common atypical CT findings (Fig. 1).

The article "Radiological findings in low-dose CT for COVID-19 pneumonia in 182 patients: Correlation of signs and severity with patient outcome" was published in 2022. Journal: Medicine (Baltimore).

Consolidation, air bronchogram, crazy paving, and pleural effusion were considered an indication of disease progression in earlier studies.^[1]^ Multivariate statistical analysis only confirmed a higher age, a higher total visual severity score, and the presence of crazy paving as predictive parameters for patient outcome and a higher total visual severity score and the presence of pleural effusion as predictive parameters for a longer hospitalization duration. Pleural effusion can be a sign of superimposed bacterial pneumonia or heart failure, as preexisting comorbidity or secondary to COVID-19 myocardial injury or COVID-19 associated pulmonary embolism.^[3–12]^ Air bronchogram, bronchial wall thickening, and enlarged lymph nodes showed a tendency to be a prognostic factor, but there is no significant correlation for patient outcome or hospital duration. The presence of an air bronchogram is a not specific sign and can be seen in other various pathologies. Enlarged lymph nodes and bronchial wall thickening are likely to be both a sign of bacterial coinfection or underlying comorbidity (e.g., COPD/emphysema and cardiac strain) rather than specific signs for COVID-pneumonia. This could be an explanation for the detected worse patient outcome and longer hospital duration in patient with these signs.

### 4.1 Biases and limitations

As mentioned above, the patient cohort consists of (mostly elderly) patients with a more severe grade of COVID-19 pneumonia and a higher need for hospital admission because of clinical deterioration. Asymptomatic and clinically less severe affected patients (usually younger patients) did not receive RT-PCR and chest CT. Furthermore, other pulmonary or chronic diseases (e.g., diabetes, chronic obstructive pulmonary disease, chronic kidney disease, immunocompromised state, etc.) that are highly related to worse COVID-19 clinical symptoms are not included in the patient characteristics.

The retrospective study used the personal CT evaluation of 4 experienced thoracic radiologists. Deep learning-based software has the potential to reduce the subjective factor by providing corrective measurements of the lung injury instead of a visual estimated severity score. Even more, there are no reliable thresholds in the evaluation of bronchial wall thickening and vascular dilatation so it is predominantly a subjective assessment on a low-dose chest CT scan.

The article "Radiological findings in low-dose CT for COVID-19 pneumonia in 182 patients: Correlation of signs and severity with patient outcome" was published in 2022. Journal: Medicine (Baltimore).

The study cohort included patients during the endemic period of COVID-19 infection in Belgium. We would like to confirm the low degree of false negatives and the high predictive value of Chest CT for COVID-19 infection when the virus is still circulating in a small amount of people and during yearly periods when seasonal flu and other respiratory infections are more common.

The study was conducted in one institution with a uniform clinical policy of the triage process based on CT examination and clinical parameters. Thanks to this policy, the availability of critical care beds was always sufficient enough during this period.

## 5 Conclusion

Chest CT scan is useful in diagnosis and triage of patients, respectively, based on the appearance of typical and atypical chest CT findings in COVID-19 pneumonia and their predictive value on patient outcome and hospital duration.

The higher predictive value of chest CT for COVID-19 infection as well as the lower degree of false negatives compared with RT-PCR makes chest CT a useful diagnostic tool. However, the study cohort included patients during the endemic period of COVID-19 infection in Belgium. So we would like to confirm these results when the pretest probability is low (in a nonendemic situation and when other viruses are circulating as well).

An increasing percentage of lung opacity as well as the presence of crazy paving and a higher age are associated with a worse patient outcome. The presence of a higher total visual severity score and pleural effusion are significant predictors for a longer hospitalization duration. Pleural effusion, considered an atypical CT finding of COVID-19 pneumonia, turned out to be predictive for a worse outcome; this is likely to be explained by superimposed bacterial pneumonia or heart failure. Even more, enlarged lymph nodes and bronchial wall thickening had a tendency to predict a worse patient outcome and longer hospital duration (significant in univariate analysis, but not enough in multivariate analysis); they are both possible signs of bacterial coinfection or underlying comorbidity (e.g., COPD/emphysema or cardiac strain) rather than typical signs of COVID-19 pneumonia. In this regard, a quick quantifiable evaluation of the lung injury (by means of a visual scoring system or deep learning based software) as well as visual screening for the presence of crazy paving and signs of bacterial coinfection or underlying comorbidity (e.g., COPD/emphysema or heart failure) can play an important role in the triage of patients with COVID-19 pneumonia to preserve the availability of critical care beds only for the patients with suspected worse outcome This quite large study gives an accurate representation to predict which patients will have a deteriorating clinical status and will need intensive care. However, additional studies are needed with deep learning based software to reduce the potential subjective factor by providing corrective measurements of the lung injury instead of a visual estimated severity score.

The article "Radiological findings in low-dose CT for COVID-19 pneumonia in 182 patients: Correlation of signs and severity with patient outcome" was published in 2022. Journal: Medicine (Baltimore).

## Author contributions

**Conceptualization:** Charlotte M. BiebaÛ, Adriana Dubbeldam.

**Data curation:** Charlotte M. BiebaÛ, Jeroen N. Desmet.

**Formal analysis:** Charlotte M. BiebaÛ, Lesley Cockmartin.

**Investigation:** Charlotte M. BiebaÛ.

**Methodology:** Charlotte M. BiebaÛ, Lesley Cockmartin.

**Project administration:** Charlotte M. BiebaÛ, Adriana Dubbeldam, Walter M. Coudyzer, Walter De Wever.

**Resources:** Charlotte M. BiebaÛ.

**Software:** Charlotte M. BiebaÛ, Walter M. Coudyzer.

**Supervision:** Adriana Dubbeldam, Johan Coolen, Johny A. Verschakelen, Walter De Wever.

**Validation:** Adriana Dubbeldam, Lesley Cockmartin, Walter De Wever.

**Visualization:** Charlotte M. BiebaÛ.

**Writing – original draft:** Charlotte M. BiebaÛ.

**Writing – review & editing:** Jeroen N. Desmet, Adriana Dubbeldam, Lesley Cockmartin, Walter M. Coudyzer, Johan Coolen, Johny A. Verschakelen, Walter De Wever.
